# Resveratrol Ameliorates Motor Neuron Degeneration and Improves Survival in SOD1^G93A^ Mouse Model of Amyotrophic Lateral Sclerosis

**DOI:** 10.1155/2014/483501

**Published:** 2014-06-26

**Authors:** Lin Song, Liang Chen, Xiaojie Zhang, Jia Li, Weidong Le

**Affiliations:** ^1^Institute of Neurology, Ruijin Hospital, Shanghai Jiao Tong University School of Medicine, Ruijin 2nd Road No. 197, Building 11-1201, Shanghai 200025, China; ^2^The Key Laboratory of Stem Cell Biology, Institute of Health Sciences, Shanghai Institutes for Biological Sciences, Chinese Academy of Sciences and Shanghai Jiao Tong University School of Medicine, Shanghai 200025, China; ^2^Center for Translational Research of Neurology Disease, First Affiliated Hospital of Dalian Medical University, Dalian 116011, China

## Abstract

Resveratrol has recently been used as a supplemental treatment for several neurological and nonneurological diseases. It is not known whether resveratrol has neuroprotective effect on amyotrophic lateral sclerosis (ALS). To assess the effect of resveratrol on the disease, we tested this agent on an ALS model of SOD1^G93A^ transgenic mouse. Rotarod measurement was performed to measure the motor function of the ALS mice. Nissl staining and SMI-32 immunofluorescent staining were used to determine motor neurons survival in the spinal cord of the ALS mice. Hematoxylin-eosin (H&E), succinic dehydrogenase (SDH), and cytochrome oxidase (COX) staining were applied to pathologically analyze the skeletal muscles of the ALS mice. We found that resveratrol treatment significantly delayed the disease onset and prolonged the lifespan of the ALS mice. Furthermore, resveratrol treatment attenuated motor neuron loss, relieved muscle atrophy, and improved mitochondrial function of muscle fibers in the ALS mice. In addition, we demonstrated that resveratrol exerted these neuroprotective effects mainly through increasing the expression of Sirt1, consequently suppressing oxidative stress and downregulating p53 and its related apoptotic pathway. Collectively, our findings suggest that resveratrol might provide a promising therapeutic intervention for ALS.

## 1. Introduction

Amyotrophic lateral sclerosis (ALS) is a progressive and fatal neurodegenerative disease, characterized by selective degeneration and death of central and peripheral motor neurons [1]. Mutations in copper/zinc superoxide dismutase (SOD1) consist of 20% cases of familial ALS (fALS), but the underlying pathogenetic mechanisms in this form of ALS are still largely unknown [2]. Our previous studies have shown a significant elevated homocysteine level in the spinal cord and serum of SOD1^G93A^ mouse model of ALS [3], and application of high dose folic acid may have therapeutic potential for the treatment of the disease [4]. We have also found that autophagy activity is increased in the spinal cord of ALS mice, pointing towards a possible role of autophagy in the pathogenesis of ALS [5]. Currently, there is no effective treatment available for ALS. Therefore, development of novel therapeutic drugs for this devastating disease is in great need.

Resveratrol (3,5,4′-trihydroxy-trans-stilbene) has received considerable attention recently for its potential neuroprotective effects in several neurodegenerative disorders [6]. But there is limited report about the application of resveratrol in ALS. Resveratrol is a polyphenolic compound present in a large number of plant species.

The direct molecular targets of resveratrol* in vitro* and* in vivo* are unknown, but it has been suggested to modulate cellular processes by regulating the expression or posttranscriptional modification of Sirtuin1 (Sirt1) and its substrates peroxisome proliferator-activated receptor-*γ* coactivator-1*α* (PGC-1*α*) and p53 [7–11]. Sirt1 is a NAD-dependent class III histone deacetylase, which resides mainly in the cell nucleus and targets several histone and nonhistone transcriptional regulators, regulating energy metabolism, cell apoptosis, protein homeostasis, and inflammation [6]. PGC-1*α* is a potent stimulator of mitochondrial biogenesis and respiration. In recent years, the role of PGC-1*α* in reactive oxygen species (ROS) metabolism and neurodegenerative diseases has been attracting great attention [12]. The tumor suppressor p53 is activated mainly through posttranslation modifications, including phosphorylation and acetylation. Lysine 382 of p53 (K382-p53) is a well-characterized target for Sirt1 deacetylase activity [6, 12]. Accordingly, we speculate that the activation of Sirt1 by resveratrol might provide neuroprotection in ALS through the suppression of the p53 acetylation and its down-stream pathway.

In the current study, we tested the neuroprotective effects of resveratrol in the SOD1^G93A^ mouse of ALS model and determined the activation of Sirt1 and its substrates as a potential underlying mechanism in ALS.

## 2. Materials and Methods

### 2.1. Animals

All the animal experiments were carried out in accordance with the guidelines laid down by the NIH in the USA regarding the care and use of animals for experimental procedures and met with ethical standards approved by the Animal Committee of Shanghai Jiaotong University School of Medicine. All efforts were made to reduce the number of animals used and to minimize animal suffering. We used SOD1^G93A^ transgenic mice, a classic animal model of ALS, in our study. The SOD1^G93A^ transgenic mice were obtained from Jackson's laboratory (number 002726). These mice usually became paralyzed in one or more limbs at approximately 90 days of age and were moribund about 30 days later [13]. The SOD1^G93A^ mice were maintained as hemizygotes by crossing transgenic male with wild-type (WT) females of the same B6SJL genetic background.

### 2.2. Intervention

To assess the effects of resveratrol on the disease onset and survival of ALS mouse model, resveratrol (Sigma; USA) was dissolved into ethanol at 50 mg/mL and further diluted with PBS at 1 : 4 (v/v) before intraperitoneal injection. Twenty male SOD1^G93A^ transgenic mice were randomly divided into two groups: (1) the resveratrol-treated group was intraperitoneally injected with resveratrol at the dose of 25 mg/kg body weight/day (*n* = 10) and (2) the vehicle-treated group, used as control, was intraperitoneally injected with the same dose of vehicle (*n* = 10). The injection was given once a day starting from the 42 days after birth until the day of the animals' death.

To explore the mechanisms of neuroprotection provided by resveratrol, 10 male SOD1^G93A^ mice and 10 age-matched WT littermates were randomly divided into four groups: resveratrol treatment at the dose of 25 mg/kg body weight/day in SOD1^G93A^ transgenic mice (Tg-RSV mice, *n* = 5) or in WT littermates (WT-RSV mice, *n* = 5) and vehicle treatment in SOD1^G93A^ transgenic mice (Tg-Veh mice, *n* = 5) or in WT littermates (WT-Veh mice, *n* = 5). They were intraperitoneally injected once a day from 42 days after birth and were sacrificed at the age of 120 days, when we collected the blood, muscle, and spinal cord tissues for biochemical and histological assays.

### 2.3. Behavioral Tests

#### 2.3.1. Assessment of Disease Onset

We started to test the rotarod performance when the mice were at the age of 70 days. The rotarod performance was examined every other day to determine the time period that the mice remained on the rotating rod (4 cm diameter, 20 rpm). When the mouse could not stay on the rotarod for 5 minutes, it was defined as the date of disease onset [14].

#### 2.3.2. Assessment of Lifespan

The mice were sacrificed, if they could not right themselves within 30 seconds being placed on a flat surface and the data was recorded as the age of death [15].

### 2.4. Pathological Analysis of Skeletal Muscles

Biopsied gastrocnemius muscles (5 × 5 × 10 mm^3^) were dissected out from the right leg of an anaesthetized animal and immersed immediately in isopentane cooled in liquid nitrogen. Serial cryostat sections were cut at 10 *μ*m and stained by hematoxylin and eosin (H&E). In addition, mitochondrial function was demonstrated by succinic dehydrogenase (SDH) staining and cytochrome oxidase (COX) staining [16].

### 2.5. Biochemical Analysis of Blood Samples

#### 2.5.1. Preparation of Blood Samples

Under deep anesthesia, blood (200 *μ*L per mouse) was collected from the eyeballs of mice at the age of 120 days. The blood was centrifuged at 4°C for 10 min at 3,000 rpm to separate the serum samples.

#### 2.5.2. Lipid Peroxidation Assay

For lipid peroxidation assay, we used a commercial kit (S0131; Beyotime; China) to measure the concentration of malondialdehyde (MDA) in spinal cord tissues and serum samples according to the manual instruction provided by the company.

### 2.6. Histopathological Analysis of Motor Neurons in Lumbar Spinal Cord

The mice were anesthetized and perfused transcardially with phosphate buffered saline (PBS) at the age of 120 days. For histopathological analysis, the spinal cord (L4-5) was removed, postfixed, and dehydrated in 15% and 30% sucrose each for 24 hours. For western blot assay, the spinal cord (C1-L3) was quickly removed and preserved in liquid nitrogen for further analysis.

The lumbar spinal cords (L4-5) were transversely sectioned at 10 *μ*m with a Leica cryostat. A total of 250 serial sections in each mouse were cut on gelatin coated slides and frozen at −80°C until use.

For immunofluorescence assay, transverse cryosections were blocked and incubated overnight at 4°C with a mouse monoclonal antibody against nonphosphorylated neurofilament H (SMI-32; 1 : 1500; Covance; USA). Then, sections were thoroughly washed and incubated for 2 hours at room temperature with the fluorescent-conjugated antibody. Fluorescence images were taken by an inverted fluorescent microscope (Olympus IX81; Japan).

For Nissl staining, every 5th section was selected from the serial sections to have 50 sections in each mouse to be stained with 1% toluidine blue at 55°C for 2 minutes. Both sides of motor neurons located in the anterior horn, which had a maximum diameter no less than 20 *μ*m and contained a distinct nucleus, were counted by investigators in a blinded manner [17].

### 2.7. Western Blotting

Fresh spinal cord tissues were dissolved and homogenized in RIPA lysis buffer containing 1% protease inhibitor phenylmethanesulfonyl fluoride (PMSF) (Sangon Biotech; China). Proteins were loaded and separated in SDS-PAGE gel and then transferred to polyvinylidene fluoride membranes. After being blocked, membranes were incubated at 4°C overnight with the following antibodies: anti-Sirt1 (1 : 1000; Santa Cruz; USA), anti-PGC1-*α* (1 : 200; Santa Cruz; USA), anti-p53 (1 : 1000; Cell Signaling; USA), anti-acetyl-p53 (1 : 1000; Millipore; USA), anti-Bax (1 : 1000; Cell Signaling; USA), anti-Bcl-2 (1 : 1000; Cell Signaling; USA), anti-caspase-3 (1 : 1000; Cell Signaling; USA), anti-Cytochrome C (Cyt C) (1 : 4000; Abcam; USA), and anti-PARP (1 : 1000; Santa Cruz; USA). After being washed thoroughly, the membranes were incubated with the appropriate secondary antibody for 2 hours. Protein bands were visualized by ECL (Pierce; USA) and an image analyzer (Quantity One-4.2.0; Bio-Rad; USA) was used to quantify the density of interested bands.

### 2.8. Statistics

SPSS 17.0 was used for statistical calculations. Disease onset and survival statistics were performed by Kaplan-Meier survival curves and the data were analyzed using the log-rank test, generating a *χ* ^2^ value to test for significance. Other data in different groups of animals were assessed by a one-way analysis of variance (ANOVA). Results were expressed as means ± SEM values.* P* values less than 0.05 were considered significant.

## 3. Results

### 3.1. Resveratrol Delayed Disease Onset and Extended the Lifespan in the SOD1^G93A^ Mice

SOD1^G93A^ transgenic mice treated with resveratrol showed significant delay of disease onset compared with vehicle-treated transgenic mice (103.40 ± 5.42 versus 92.20 ± 4.64 days, *χ* ^2^ = 11.16, *P* < 0.01) (Figure 1(a)). The lifespan of SOD1^G93A^ mice treated with resveratrol was 14.40 days longer than the vehicle-treated counterparts (136.80 ± 9.02 versus 122.40 ± 9.63 days, *χ* ^2^ = 8.29, *P* < 0.01) (Figure 1(b)).

### 3.2. Resveratrol Ameliorated Motor Neuron Loss in the SOD1^G93A^ Mice

From the immunofluorescence images, motor neurons in the anterior horn of lumbar spinal cord in Tg-Veh mice were fewer and smaller than those of the WT-Veh mice, while resveratrol treatment significantly protected the motor neurons in the Tg-RSV mice (Figure 2(a)). We then quantitatively counted in a blind manner the number of Nissl's stained-motor neurons. Compared with the WT-Veh littermates, only 33.19% of the motor neurons remained at the same level of the spinal cord in the Tg-Veh mice (264.25 ± 21.25 versus 796.25 ± 42.61, *P* < 0.001). However, resveratrol injection in the Tg-RSV mice retained 81.48% of the motor neurons compared with the Tg-Veh mice (438.75 ± 41.31 versus 796.25 ± 42.61, *P* < 0.01). No significant difference was found between the WT-RSV and WT-Veh mice (811.75 ± 50.20 versus 796.25 ± 42.61, *P* > 0.05) (Figures 2(b) and 2(c)).

### 3.3. Resveratrol Ameliorated the Atrophy and Mitochondrial Dysfunction in the Muscle Fibers of SOD1^G93A^ Mice

Using H&E staining, we found that the ALS mice treated with vehicle showed significant reduction in cross-section area of gastrocnemius muscle fibers compared with their age-matched WT-Veh littermates. Resveratrol administration increased the cross-section area gastrocnemius muscle fibers in the Tg-RSV mice compared with the Tg-Veh counterparts (Figure 3). We did not find central nuclei in the Tg-RSV mice (Figure 3).

SDH staining is regarded as the standard screening reaction for mitochondria [14]. Notably, the SDH staining of the metabolic activity of skeletal muscles showed a high level of oxidative stress in the Tg-Veh mice as compared with the WT-Veh littermates (Figure 3). However, the increase of SDH staining was significantly attenuated in the resveratrol-injected Tg-RSV mice.

COX is another mitochondrial enzyme, which reflects the capacity of cells to undergo mitochondrial electron transport and oxidative phosphorylation [18]. We observed that, in the Tg-Veh mice, some muscle fibers had no staining for COX. The deficiency of COX may indicate the overproduction of ROS, which renders the mitochondrial genome susceptible to ROS-induced injury. However, in the Tg-RSV mice, it seemed that most of the muscle fibers were COX positive.

### 3.4. Resveratrol Regulated the Expression of Sirt1 and PGC1-*α* and Improved the Lipid Peroxidation in the SOD1^G93A^ Mice

The level of Sirt1 in the Tg-Veh mice was nearly half as seen in the WT-Veh mice (0.98 ± 0.09 versus 1.91 ± 0.15, *P* < 0.01). After the chronic treatment with resveratrol, the Sirt1 levels in the spinal cords of Tg-RSV and WT-RSV mice were increased by 49.22% and 47.96%, respectively (1.46 ± 0.09 versus 0.98 ± 0.09, *P* < 0.05 and 2.85 ± 0.19 versus 1.91 ± 0.15, *P* < 0.01) (Figures 4(a) and 4(c)). Further, we found that PGC-1*α* level in the spinal cords of Tg-Veh mice was increased up to 276.42% compared with the WT-Veh littermates, whereas resveratrol administration significantly suppressed the expression of PGC-1*α*, making it near the level of WT-Veh littermates. There was no significant difference of PGC-1*α* between WT-Veh and WT-RSV mice (Figures 4(b) and 4(d)).

In the Tg-Veh mice, the level of MDA was nearly 4-fold that in the WT-Veh mice (20.30 ± 2.16 versus 5.88 ± 1.32 *μ*mol/L, *P* < 0.001), whereas resveratrol treatment significantly decreased the MDA level by 33.70% in the ALS mice (13.46 ± 1.29 versus 20.30 ± 2.16, *P* < 0.01). Similarly, in the spinal cords of Tg-RSV mice, the MDA level was moderately lower than that in the Tg-Veh mice, although the statistical analysis showed no significant difference.

### 3.5. Resveratrol Inhibited p53 and Its Downstream Apoptotic Pathway in the ALS Mice

The quantitative analysis showed that the level of p53 in the Tg-Veh mice was nearly 4-fold that in the WT-Veh mice. The level of p53 was decreased by 58.80% after the resveratrol treatment in the Tg-RSV mice (1.71 ± 0.24 versus 4.15 ± 0.27, *P* < 0.001). Similarly, the level of acetyl-p53 in the Tg-Veh mice was 74.04% higher than that of the WT-Veh mice (1.81 ± 0.07 versus 1.04 ± 0.14, *P* < 0.01) but was decreased by 20.99% after the resveratrol treatment (1.43 ± 0.09 versus 1.81 ± 0.07, *P* < 0.05).

We then determined the mitochondria-dependent apoptosis protein levels of Bax, Bcl-2, cleaved caspase-3, Cyt C, and cleaved PARP. The Western blot results showed that the antiapoptotic protein level of Bcl-2 was considerably reduced in the Tg-Veh mice compared with the WT-Veh mice, while resveratrol treatment in the Tg-RSV mice increased the level of Bcl-2. Conversely, Bax, cleaved caspase-3, Cyt C, and cleaved PARP were markedly elevated in the Tg-Veh mice, and resveratrol administration could suppress the expression of these proteins in the Tg-RSV mice. However, all of the apoptosis-related molecules were not affected in the WT-RSV mice compared with the WT-Veh mice (Figure 5(B)).

## 4. Discussion

Our study provides first evidence that resveratrol treatment can delay the onset of disease and prolong the lifespan in a well-established ALS mouse model, probably through the protection of motor neurons and skeletal muscles. The neuroprotective effects of resveratrol may be related to its biological role to increase the expression of Sirt1, suppress the expression of PGC-1*α*, and inhibit oxidative stress in the spinal cord of the ALS mice. Furthermore, resveratrol has significant antiapoptotic effects by upregulating Bcl-2 and inhibiting p53 and its downstream apoptotic pathway.

Resveratrol has been one of the most extensively studied polyphenols recently owing to its potent therapeutic activities. However, the* in vivo* biological effects of resveratrol appear strongly limited by its low bioavailability [19]. In the present study, we put our efforts to improve its bioavailability. Firstly, reseratrol was kept away from light, since it is an extremely photosensitive compound. In addition, we used 10% ethanol in PBS as vehicle to enhance the solubility of resveratrol. Moreover, we gave the solution through interperitioneal injection, reducing the first pass effect.

Oxidative stress and mitochondrial dysfunction have been regarded as important risk factors for pathogenesis of ALS [20, 21]. It was reported that resveratrol could improve mitochondrial function and protect against metabolic disease by activating Sirt1 and PGC-1*α* in C57B1/6J mice [22]. In this study, we found that resveratrol also activated Sirt1 and improved mitochondrial function in the ALS mice. MDA, which reflects the severity of oxidative stress, was significantly decreased in the sera and in the spinal cords of Tg-RSV mice compared with the Tg-Veh mice. We considered that the antioxidant effect of resveratrol resulted partly, at least, from the activation of Sirt1.

Previous works reported that the expression of PGC-1*α* was regulated by Sirt1 in different tissues [23, 24]. Overexpression of PGC-1*α* could significantly improve motor function and prolong the lifespan of ALS mice, which indicate that PGC-1*α* may play a protective role in ALS [25]. Moreover, it has been suggested that AMPK, p38 MARK, and ROS were involved in the regulation of PGC-1*α* [11, 26]. PGC-1*α* can be induced by elevated ROS as a responsive protective effort in neural cells [27]. In our study, we found that the level of PGC-1*α* was dramatically increased in Tg-Veh mice compared with WT-Veh or WT-RSV mice, indicating that the elevated ROS might be involved in the increase of PGC-1*α* in the ALS mice (Figure 4(a)). We also demonstrated that the level of ROS was suppressed after the resveratrol treatment (Figures 4(e) and 4(f)), and then the level of PGC-1*α* was significantly reduced (Figure 4(a)) which we believe that it might be the result of the decreased ROS level in Tg-RSV mice.

Increasing evidences support that apoptosis activation is the terminal process of motor neuron death in ALS [28]. p53 can bind to Bcl-2 and thus promote opening of the mitochondrial pore with mitochondrial permeabilization, release of cytochrome* c*, and activation of caspase-3 and leads to apoptotic cell death [1]. p53 is a sequence-specific transcription factor that is dramatically increased in response to a variety of cellular stresses, and its activation may cause cell death by directly inducing mitochondrial permeability and apoptosis [3, 29]. Now, Sirt1 is believed to regulate apoptotic thresholds by deacetylating p53 [6, 12]. In our study, we documented that resveratrol can have neuroprotective effect through the Sirtl mediated anti-p53 apoptotic pathway in the ALS mice.

Aberrant protein misfolding is known to contribute to the pathogenesis of ALS and possibly is related to the defect of autophagy-lysosomal pathway, which may exacerbate the pathological processing through apoptotic and other mechanisms in the disease [30]. We confirm in our study that the strong inhibition effects of resveratrol on apoptosis through the upregulation of Bcl-2 and suppression of Bax, cleaved caspase-3, p53, and acetyl-p53 as well as its down-stream mitochondria-dependent apoptotic pathway. We believe that these collective effects prevent the motor neurons from degeneration in ALS.

## 5. Conclusions

Taken together, our findings indicate that resveratrol could delay the onset of disease and prolong the lifespan of SOD1^G93A^ mice. Resveratrol can significantly attenuate the motor neuron loss and reduce the muscle atrophy and dysfunction in the ALS mice. It is likely that the antioxidant and antiapoptotic effects of resveratrol are the major beneficial roles of this compound to play against ALS.

## Figures and Tables

**Figure 1:** The benefit effects of resveratrol on disease onset and lifespan in the SOD1^G93A^ mice. Kaplan-Meier survival curves indicated, respectively, the probability of (a) disease onset and (b) survival in the vehicle or resveratrol-treated ALS mice. *N* = 10 in each group.

**Figure 2:** Resveratrol administration prevented motor neuron death in SOD1^G93A^ mice at the age of 120 days. (a) Immunofluorescent staining of motor neurons (white arrows) with SMI-32 (green) antibody in the anterior horn of spinal cord from different groups of mice. (b) Photomicrographs of Nissl's stained-motor neurons (black arrows) in the anterior horn of the spinal cord of SOD1^G93A^ mice in different groups. (A) WT-Veh group, (B) WT-RSV group, (C) Tg-Veh group, and (D) Tg-RSV group. (c) Quantification of motor neurons in the anterior horn of lumbar spinal cord in different groups. The values are means ± SEM. ^##^ *P* < 0.001 versus WT-Veh group; *P < 0.01 versus Tg-Veh group; ^&&^ *P* < 0.001 versus Tg-RSV group. *N* = 5 in each group. Scale bar = 100 *μ*m.

**Figure 3:** Effects of resveratrol on the gastrocnemius muscles from different groups of mice at the age of 120 days. Black arrows indicated the myofibers with internal myonuclei; white arrows indicated myofibers with absent COX staining.

**Figure 4:** Effects of resveratrol on oxidative capacity in different groups of mice. (a) Western blot assay of Sirt1 and PGC1-*α* in the spinal cord tissues of WT and transgenic mice treated or untreated with resveratrol. (b) Relative Sirt1 mRNA expression in the spinal cords of different groups of mice. (c-d) Quantitative analysis of the protein expression of (c) SIRT1 and (d) PGC1-*α* in the spinal cords. (e-f) MDA concentration in (e) serum and (f) spinal cords from different groups of mice. The values are means ± SEM. ^#^ *P* < 0.01 and ^##^ *P* < 0.001 versus WT-Veh group; *P < 0.01 and **P < 0.001 versus Tg-Veh group; ^&^ *P* < 0.01 and ^&&^ *P* < 0.001 versus Tg-RSV group. *N* = 5 in each group.

**Figure 5:** Expression of apoptosis-related molecules in WT and transgenic mice treated with vehicle or resveratrol. (A–F) Western blot assay of (A) p53, (B) acetyl-p53, (C) Bax/Bcl-2, (D) cleaved caspase-3, (E) Cyt C, and (F) PARP from the spinal cord tissues in different groups of mice. (a–f) Quantitative data of the expression of (a) p53, (b) acetyl-p53, (c) Bax/Bcl-2, (d) cleaved caspase-3, (e) Cyt C, and (f) PARP in the four groups of mice. The values are means ± SEM. ^##^ *P* < 0.01 and ^###^ *P* < 0.001 versus WT-Veh group; *P < 0.05, **P < 0.01, and ***P < 0.001 versus Tg-Veh group; ^&^ *P* < 0.05 and ^&&^ *P* < 0.01 versus Tg-RSV group. *N* = 5 in each group.

## Abbreviations

ALS: Amyotrophic lateral sclerosis
COX: Cytochrome oxidase
Cyt C: Cytochrome C
H&E: Hematoxylin and eosin
MD: Malondialdehyde
PBS: Phosphate buffered saline
PGC1-*α*: Peroxisome proliferator-activated receptor-*γ* coactivator-1*α*
PMSF: Phenylmethanesulfonyl fluoride
ROS: Reactive oxygen species
SDH: Succinic dehydrogenase
Sirt1: Sirtuin1
SMI-32: Nonphosphorylated neurofilament
SOD1: Copper/zinc superoxide dismutase
WT: Wild-type.
